The article "Crosstalk between autophagy and metabolic regulation of cancer stem cells" was published in 2020. Journal: Mol Cancer.

# Crosstalk between autophagy and metabolic regulation of cancer stem cells

**DOI:** 10.1186/s12943-019-1126-8

**Published:** 2020-02-06

**Authors:** Mouradi El Hout, Emma Cosialls, Maryam Mehrpour, Ahmed Hamaï

**Affiliations:** 1 Institut Necker-Enfants Malades (INEM), Inserm U1151-CNRS UMR 8253, F-75993 Paris, France; 2 Université Paris Descartes-Sorbonne Paris Cité, F-75993 Paris, France

**Keywords:** Cancer stem cells, Autophagy, Metabolic heterogeneity, Lipid metabolism, Therapeutic target

## Abstract

Cancer is now considered as a heterogeneous ecosystem in which tumor cells collaborate with each other and with host cells in their microenvironment. As circumstances change, the ecosystem evolves to ensure the survival and growth of the cancer cells. In this ecosystem, metabolism is not only a key player but also drives stemness. In this review, we first summarize our current understanding of how autophagy influences cancer stem cell phenotype. We emphasize metabolic pathways in cancer stem cells and discuss how autophagy-mediated regulation metabolism is involved in their maintenance and proliferation. We then provide an update on the role of metabolic reprogramming and plasticity in cancer stem cells. Finally, we discuss how metabolic pathways in cancer stem cells could be therapeutically targeted.

## Background

Cancer is a heterogeneous disease, and metabolic flexibility of tumors contributes to this heterogeneity. As circumstances change, the tumor ecosystem evolves to ensure the survival and growth of the cancer cells [1]. In this ecosystem, metabolism is a driver of stemness [2]. Cancer stem cells (CSCs) are a subset of cells within tumors that have the capacity to generate tumors and that exhibit self-renewal and differentiation properties. CSCs are resistant to cancer therapies and are a distinct population associated with metastasis and relapse.

Only a few studies have directly examined the metabolism of CSCs in large part due to difficulties in isolating this population. Currently, there are more than 40 established CSC markers; however, most are also present in human embryonic stem cells and/or adult stem cells from normal tissues and a consensus marker for the identification of CSCs still a matter of debate. We begin this review with a brief discussion of autophagy and CSCs, and we review recent data on CSC metabolism. Finally, we discuss how CSC metabolism could be a therapeutic target for treatment of cancer.

## Autophagy in CSCs

Autophagy is a process necessary for normal cellular function involved in the tumor initiation, tumor interactions with neighboring cells in the tumor microenvironment, and cancer therapy. The role of autophagy in cancer is multifaceted: Autophagy promotes tumor cell survival by supplying recycled metabolites for growth, modulates mitochondrial function via mitophagy (the selective degradation of mitochondria), and functions in tumor cell migration and invasion via control of secretion of pro-migratory cytokines and focal adhesion turnover [3]. Also, several studies have demonstrated that autophagy plays a central role in the tumor microenvironment [3, 4]. For example, autophagy is induced in cancer-associated fibroblasts (CAFs) by their association with tumor cells, and this results in increased fibroblast production of amino acids, which are provided in a paracrine manner to tumor cells to sustain their growth [5]. Two important elements that influence metabolic reprogramming of tumors are their microenvironment and the distance to the vasculature [1, 4]. First, emerging evidence indicates the unexpected ability of malignant cells (both CSCs and non-CSCs) to supplement their metabolism with nutrients provided by neighboring cells with complementary metabolic activities, enhancing tumor cell survival and proliferative capacity [6–8]. Second, cancer cells located closer to the blood supply generate ATP via oxidative stress, and this induces glycolysis and autophagy in the surrounding catabolic stromal/cancer cells (again, in both CSCs and non-CSCs), which generate catabolites such as fatty acids, lactates, and ketones that in turn are taken up by anabolic cancer cells (both CSCs and non-CSCs) and used to fuel mitochondrial metabolism and ATP production. This is known as the reverse Warburg effect (Table 1). Parallel autophagic responses activated in distal and poorly oxygenated tumor areas provide catabolic intermediates to sustain anabolic demands and support cancer growth (Table 1).

The article "Crosstalk between autophagy and metabolic regulation of cancer stem cells" was published in 2020. Journal: Mol Cancer.

**Table 1:** Warburg and Reverse Warburg effects

Aerobic glycolysis, or the Warburg effect, is a phenomenon in cancer cells that results in reorientation of metabolism to the glycolytic pathway and to conversion of pyruvate resulting from glycolysis into lactate even in the presence of oxygen. This metabolic reprogramming is a step in the process of tumorigenesis in many cancers. It is one of the best-described metabolic adaptations arising in cancer cells. It is now established, however, that malignant transformation is not based solely on the Warburg effect. Indeed, tumor cells produce a significant fraction of their ATP via oxidative phosphorylation (OXPHOS). Malignant cells adapt their energetic metabolism to the conditions of the microenvironment, in particular to the oxygenation conditions of the tumor, which has the consequence of creating intra-tumor metabolic heterogeneity (for additional information see [1, 9, 10]). The reverse Warburg effect is observed when anabolic epithelial cancer cells induce aerobic glycolysis in neighboring stromal fibroblasts or neighboring catabolic cancer cells. These catabolic cells (epithelial cancer cells or cancer-associated fibroblasts) secrete catabolites such as lactate, pyruvate (energy metabolites resulting from aerobic glycolysis), free fatty acids, and ketone bodies. Anabolic epithelial cancer cells take up these energy-rich metabolites and use them to fuel OXPHOS. This results in a higher proliferative capacity (see Fig. 1 and [1]). An absence of stromal Cav-1 may be a biomarker for the reverse Warburg effect.	

Recent reviews have focused on the role of autophagy in tumor metabolism [4], anti-tumor immunity [3], and cancer metastasis and cancer therapy [11]. Here, we briefly discuss more recently reported roles for autophagy in CSCs. Autophagy appears to be necessary for the maintenance of stemness in both normal tissue stem cells [12] and CSCs [13, 14] in diverse cancer types including breast, pancreatic, bladder, and colorectal cancers, chronic myeloid leukemia, and glioblastoma (for review see [8]). The survival and quiescence of normal tissue stem cells is dependent on autophagy, and autophagy has also been reported to promote pluripotency. In CSCs, autophagy promotes expression of stem cell markers such as CD44 as well as expression of mesenchymal markers such as vimentin [13]. Autophagy also promotes spheroid formation in vivo tumorigenesis consistent with a critical role in maintaining CSCs [14]. Further, the inhibition of autophagy limits tumor dormancy and promotes outgrowth of metastases [15]. Key transcription factors have been linked to the induction of autophagy and the stem cell state including Forkhead box 3A (FOXO3A), which induces expression of autophagy genes in stem cells and is itself turned over by autophagy. Other transcription factors, including the core stemness factors sex determining region Y-box (SOX2) and Nanog Homeobox (NANOG), have also been linked to autophagy induction [16]. Also, SOX2 and STAT3 have been shown to modulate autophagy genes and to determine the stemness of CSCs.

Mitophagy is emerging as a key in the control of normal tissue stem cell homeostasis. Mitophagy functions to control mitochondria quality and also regulates cellular metabolism. For example, removing damaged mitochondria, the main source of ROS, by mitophagy prevents senescence and limits ROS-induced genome damage. Limiting ROS damage is essential for maintenance of stemness. An essential role for mitophagy has reported during the glycolytic switch necessary for mouse developmental neurogenesis [12]. The turnover of mitochondria through mitophagy helps to maintain the stem cell state by limiting the capacity of the stem cells for oxidative phosphorylation (OXPHOS) and making the stem cells more dependent on glycolysis for energy demands. Inhibition of mitophagy suppresses CD44 expression and also promotes translocation of p53 to the nucleus, where it antagonizes expression of stem cell genes.

The article "Crosstalk between autophagy and metabolic regulation of cancer stem cells" was published in 2020. Journal: Mol Cancer.

The high levels of autophagy observed in CSCs are associated with the maintenance of pluripotency, with resistance to chemotherapy, and with migration and invasion [3]. Autophagy allows CSCs to survive despite hypoxia and low levels of nutrients in the tumor microenvironment [17]. Missing is a comprehensive view of how these processes drive CSC fate, and few of the regulatory molecules involved have been identified. Readers interested in detailed discussion of autophagy processes in CSCs should see a recent review [8].

## CSCs are more glycolytic than other differentiated cancer cells

A growing body of evidence suggests that the metabolism of CSC also differs from that of the bulk tumors. The importance of glucose for the maintenance and propagation of CSCs was first established in glioblastoma (GBM) [18] and then in other types of cancer including breast cancer, colon cancer, lung cancer, ovarian cancer, and osteosarcoma [2]. The side population cells with CSC characteristics avidly consume glucose and generate a significant amount of ATP and lactate [19]. In addition, in these cells the AKT Kinase pathway is activated by glucose and inhibition of glycolysis decreases the ability of these cells to form tumors in vivo. In ovarian cancer, the CD44^+^/MyD88^+^ CSCs depend only on glycolysis for their survival and are incapable of producing ATP by OXPHOS, resulting in autophagic death in the absence of glucose [20].

The metabolism of breast CSCs (BCSCs) grown as spheres is strongly associated with increased activities of key enzymes of anaerobic glucose fate such as pyruvate kinase isozyme M2 (PKM2), lactate dehydrogenase (LDH), and glucose-6-phosphate dehydrogenase (G6PDH). Consistent with this, BCSCs are highly sensitive to 2-deoxyglucose, a well-known inhibitor of glycolysis [21]. The overexpression of fructose-1,6- biphosphatase (FBP1) and the increase of ROS are accompanied by a significant reduction in the number of CD44^high^/CD24^low^/EpCAM^+^ CSCs and the formation of spheres [22]. The increase of glucose uptake, glycolytic enzyme expression, lactate production, and ATP content in CSCs compared with their differentiated counterparts seems to be linked to a concomitant reduction in mitochondrial activity [18, 21] and also to maintenance of OXPHOS and beta-oxidation [23]. Mechanistic analysis demonstrated that decreased expression and activity of pyruvate dehydrogenase (PDH), a key regulator of oxidative phosphorylation, plays a critical role in promoting the pro-glycolytic phenotype of CSCs. Metabolic reprogramming via forced activation of PDH preferentially eliminates CSCs [24]. Tamada et al. showed that CD44, a marker of CSCs, acts as a metabolic modulator, activating glycolysis under hypoxic conditions and reducing glycolysis and antioxidant responses and enhancing mitochondrial production with associated increases in ROS. CD44 interacts with PKM2 in different cancer cell lines and inhibits its activity, correlating with the glycolytic phenotypes of p53-deficient cells [25]. A metabolic signature characteristic of colon cancer initiating cells has been associated with increased expression of genes and metabolites of the glycolytic pathway and the tricarboxylic acid cycle (TCA) [26].

The article "Crosstalk between autophagy and metabolic regulation of cancer stem cells" was published in 2020. Journal: Mol Cancer.

## CSCs rely on mitochondrial oxidative metabolism

In contrast to data linking the stem phenotype of cancer cells to glycolytic metabolism, emerging evidence indicates that CSCs have a preference for OXPHOS metabolism (Fig. 1). In both cases, mitochondrial function is essential for stemness, migration, and drug resistance of CSCs [27]. Compared to differentiated progeny, BCSCs consume more glucose, produce less lactate, and have higher ATP content. BCSCs are heterogeneous in their metabolic phenotypes and have metabolic states distinct from their differentiated progeny.

**Fig. 1:** The metabolic heterogeneity of cancer stem cells. Tumors are complex and dynamic structures encompassing populations of host cells (e.g., fibroblasts and immune cells) and cancer cells with different metabolic activities. These cells are affected in different ways by microenvironmental conditions and biological activities of other tumor cells. For example, cancer cells close to the vasculature show oxidative metabolism, whereas a shift toward a glycolytic metabolism is observed when glucose is present in cells residing in hypoxic areas. Despite metabolic heterogeneity, cancer cells cooperate to allow adaption to changes in conditions to ensure that metabolic requirements are met. Indeed, oxidative cancer cells, like proliferating cells, increase the consumption of glucose to produce ATP and generate biomass to support cell proliferation. The oxidative stress caused by rapidly proliferation of cancer cells induces glycolysis and autophagy/mitophagy in stromal cells and/or in glycolytic cancer cells leading to the release of high amounts of lactate, which fuels the metabolism of oxidative cancer cells. Key elements of lactate shuttles are the plasma membrane monocarboxylate transporters. MCT4 is involved in the export of lactate, and MCT1 and MCT2 are involved in the uptake of this catabolite. High levels of several factors including HIF-1α, NF-κB, TGF-β, and JNK/AP1 are associated with glycolytic phenotype. The metabolic status of a CSC depends on location. In actively growing regions of the tumor and in the presence of adequate levels of oxygen (normoxic conditions), CSCs rely on glycolytic and/or oxidative metabolism. Overexpression of HIF-1α in the hypoxic environment promotes upregulation of GLUT1, GLUT3, and glycolytic enzymes. In the metastatic niche, CSCs have increased utilization of extracellular catabolites. In nutrient-poor states, autophagy is activated to provide an alternative energy source. OXPHOS and the anabolic gluconeogenesis pathways control glucose homeostasis. Abbreviations: ATP, adenosine triphosphate; CSC, cancer stem cell; GLUT1/GLUT3, glucose transporter 1/3; HIF-1α, hypoxia-inducible factor 1α; HK2, hexokinase 2; JNK/AP1, c-Jun N-terminal kinases/activator protein 1; LDH, Lactate dehydrogenase; XMCT2/4, monocarboxylate transporter 2/4; NF-κB, nuclear factor-κB; OXPHOS, oxidative phosphorylation; PFKFB, phosphofructokinase/fructose bisphosphate; PKM2, pyruvate kinase isozyme M2; TGF-β, transforming growth factor β

The increased mitochondrial mass in a distinct population of breast cancer cells is attributed to a stem-like phenotype and is associated with metastatic potential and chemotherapy resistance [28]. Despite a high rate of pentose phosphate pathway activity, which is not typical of cells that prefer OXPHOS over glycolysis, the CSCs isolated from patients with epithelial cancer overexpress genes associated with glucose uptake, OXPHOS, and fatty acid beta oxidation, indicating that in these cells pyruvate is preferentially directed toward the TCA cycle. Consistent with a metabolic OXPHOS profile, CSCs have higher mitochondrial ROS production and elevated membrane potential than normal cells and undergo apoptosis upon inhibition of the mitochondrial respiratory chain [29]. Consistent with previously reported data [30], CSCs display enhanced antioxidant defenses compared to their non-tumorigenic counterparts, and this may contribute to tumor resistance to therapy.

The article "Crosstalk between autophagy and metabolic regulation of cancer stem cells" was published in 2020. Journal: Mol Cancer.

De Luca et al. recently reported that mitochondrial biogenesis is required for maintenance of stem-like properties [31]. The inhibition of mitochondrial biogenesis mediator PGC1α decreases the stem-like properties of BCSCs [31]. In pancreatic ductal adenocarcinoma (PDAC), the deadliest cancer in western countries, it has been shown that CSCs are OXPHOS-dependent, unlike non-CSCs that are glycolytic. In addition, suppression of MYC expression and increased expression of PGC1α are key determinants for the OXPHOS dependency of CSCs and their limited ability to switch to glycolysis during mitochondrial inhibition [32].

A recent study showed that Matcha green tea inhibits the propagation of BCSCs. Interestingly, metabolic phenotyping revealed that treatment with this compound suppresses both OXPHOS and glycolytic flux, shifting cancer cells toward a more quiescent metabolic state [33].

## Other metabolic pathways involved in CSC maintenance and proliferation

### Mevalonate metabolic pathway

A prominent role of the mevalonate metabolic pathway in regulating the self-renewal of basal/mesenchymal BCSCs has been demonstrated. Inhibition of this pathway with hydroxy-3-methylglutaryl CoA reductase blockers results in a reduction of BCSC proliferation independent of inhibition of cholesterol biosynthesis and of protein farnesylation. Notably, geranylgeranyl transferase I is crucial for BCSC maintenance. The effect of geranylgeranyl transferase I on the CSC subpopulation is mediated by inactivation of Ras homolog family member RHOA and increased accumulation of P27^kip1^ in the nucleus [34]. Mesenchymal stem cells have been reported to shuttle mitochondria and/or mitochondrial DNA in leukemia, lung, and breast tumors and to consume the cysteine dimer cystine to provide leukemic cells with chemoprotective cysteine [7].

### Hypoxia and redox homeostasis

Clinical data indicate that reduced oxygen availability, or hypoxia, observed in intratumoral regions activates hypoxia-inducible factors (HIFs). These master regulators of oxygen homeostasis also play key roles in the maintenance of BCSCs [35]. In response to intratumoral hypoxia or chemotherapy such as carboplatin or paclitaxel, the increased expression of HIF-1α and HIF-2α in BCSCs leads to increased expression of pluripotency factors such as Kruppel-like Factor 4 (KLF4), NANOG, octamer-binding transcription factor 4 (OCT4), and SOX2 [35]. HIF-1 coordinately regulates expression of genes encoding pyruvate dehydrogenase (PHGDH) and five downstream enzymes in the serine synthesis pathway and mitochondrial one-carbon (folate) cycle. Silencing of *PHGDH* expression leads to decreased NADPH levels, disturbed mitochondrial redox homeostasis, and increased apoptosis, which abrogate BCSC enrichment under hypoxic conditions. PHGDH-deficient cells are relatively weakly tumorigenic, and tumors that do form are deficient in BCSCs and thus have no metastatic capacity [36]. Human non-small cell lung cancer cells cultured in low folate conditions have enhanced CSC-like properties associated with elevated lactate release and medium acidification, suppressed expression of PDH, and elevated redox status as shown by NADH/NAD^+^ and NADPH/NADP^+^ ratios. These data are indicative of the metabolic reprogramming to aerobic glycolysis. Genetic and pharmacological inhibition of mechanistic target of rapamycin (mTOR) abrogates low folate-activated AKT-mTOR-HIF1-FOXO3a signaling and stemness-associated sonic hedgehog pathway activity, reverses the Warburg metabolic switch, and diminishes invasiveness of non-small cell lung cancer cells. These data suggest that lung CSCs may arise from a microenvironment low in folate through the activation of an AKT-mTOR-HIF1-FOXO3a signaling network, which promotes bioenergetic reprogramming to enhance CSC-like signatures and invasion and metastasis of lung cancers [37].

The article "Crosstalk between autophagy and metabolic regulation of cancer stem cells" was published in 2020. Journal: Mol Cancer.

### NAD and nicotinamide phosphoribosyl transferase pathways are associated with tumorigenesis

NAD is a cofactor essential for metabolism, energy production, DNA repair, maintenance of mitochondrial fitness, and signaling in many types of cancer cells. The biosynthesis of NAD occurs through both de novo and salvage pathways. NAD is primarily synthesized from nicotinamide, a process known as the NAD salvage pathway. Nicotinamide phosphoribosyl transferase (NAMPT) catalyzes the conversion of nicotinamide to nicotinamide mononucleotide (NMN), which is the rate-limiting step in the NAD salvage pathway. Thus, NAMPT is critical for NAD biosynthesis. Inhibition of NAMPT leads to depletion of NAD^+^, which in turn inhibits ATP synthesis [38]. NAMPT is overexpressed in high-grade glioma and GBM tumors, and its levels correlate with tumor grade and prognosis. Ectopic overexpression of NAMPT in glioma cell lines is associated with the enrichment of glioblastoma CSC population and inhibition of NAMPT blocks in vivo tumorigenicity of glioblastoma CSCs. The self-renewal properties of the glioblastoma CSC population and radiation resistance in GBM are orchestrated by a NAD-dependent transcriptional network [39]. Along the same lines, Lucena-Cacace et al. also recently reported that NAMPT plays an important role in regulation of the CSC survival and proliferation in colon cancer tumors [40]. This phenotype is mediated by poly (ADP-ribose) polymerases (PARPs) and sirtuins (SIRTs).

Recently, Lucena-Cacace et al. raised the idea that NAMPT contributes to tumor dedifferentiation and, driven by NAD supply, is responsible for the epigenetic reprogramming observed in tumors [37]. This idea is supported by data reported by Jung et al. [41] who showed that mesenchymal glioblastoma stem cells (GSCs) contain higher levels of NAD and lower levels of nicotinamide, methionine, and S-adenosyl methionine (SAM), a methyl donor generated from methionine, compared to differentiated tumor cells. Nicotinamide N-methyltransferase (NNMT), an enzyme that catalyzes the transfer of a methyl group from the cofactor SAM onto its various substrates such as nicotinamide and other pyridines, is also overexpressed in GSCs. Increases in NNMT lead to a decrease in SAM. GSCs are hypomethylated in GBM, and this causes tumors to shift toward a mesenchymal phenotype with accelerated growth, a phenotype also associated with overexpression of NAMPT. *NNMT* silencing decreases self-renewal and in vivo tumor growth of GSCs. Inhibition of NNMT expression or activity also diminishes methyl donor availability, thus decreasing methionine and unmethylated cytosine levels. Available data suggest that NNMT has a dual mechanism: It promotes DNA hypomethylation through reduction of methyl donor availability and through downregulation of activities of DNA methyltransferases such as DNMT1 and DNMT3A [41].

The article "Crosstalk between autophagy and metabolic regulation of cancer stem cells" was published in 2020. Journal: Mol Cancer.

### NAD^+^ and autophagy

Decreased NAD^+^ availability compromises the PARP1-associated base excision DNA repair pathway. Chemical inhibition of PARP1 using the drug olaparib impairs base excision DNA repair thereby enhancing temozolomide-induced damage; this mechanism is responsible for synergistic anti-tumor effects of the two drugs in GSC lines [42]. Mechanistic studies suggest that the activation of PARP1 upregulates the AMP-activated protein kinase (AMPK) signal pathway and downregulates the mTOR signaling pathway, thereby promoting autophagy following ionizing radiation or starvation [43].

NAD^+^ consumption by PARP1 generates a Ca^2+^ mobilizing messenger and upregulates intracellular Ca^2+^ signaling through transient receptor potential melastatin 2 channels, which can also enhance autophagy. However, further studies are required to confirm that NAD^+^ metabolism induced by PARP1 contributes to autophagy initiation in CSCs. Pharmacological or genetic manipulation of NAD levels appears to modulate autophagy by altering SIRT1 activity. Inhibition of SIRT1 abolishes this autophagy modulation, suggesting that SIRT1 is critical for this process. The mechanisms underlying the NAD^+^-dependent deacetylation by SIRT1 in the regulation of autophagy involve the activation or inhibition of multiple transcription factors, including FOXO3 and P53, and of ATG proteins such as ATG5, ATG12, ATG14, Beclin-1, Bcl-2/adenovirus E1B interacting protein 3 (Bnip3), and Microtubule-associated Protein 1 Light Chain 3 (LC3) [44]. However, further studies are required to confirm that NAD^+^ metabolism regulated by SIRT1 contributes to autophagy initiation in CSCs.

The article "Crosstalk between autophagy and metabolic regulation of cancer stem cells" was published in 2020. Journal: Mol Cancer.

### Glutaminolysis

Glutaminolysis is also essential for the proliferation and survival of epithelial CSCs largely because the ammonia molecules released from glutamine metabolism neutralize the excessive levels of protons (lactic acid) that result from the marked Warburg effect observed in these cells [45]. Epithelial CSCs preferentially rely on aerobic glycolysis for bioenergetics, display an active serine-one-carbon-glycine metabolism, and show an increased metabolic flexibility to utilize different carbon sources (such as fatty acids and glutamine) that offsets the decreased diversion of glucose-derived carbons into the TCA cycle.

Recent studies have shed light on the role of iron metabolism in CSCs and suggest that specific targeting of iron metabolism in CSCs may improve the efficacy of cancer therapy. Readers interested in detailed discussion of iron metabolism in CSCs should see a recent review [46, 47].

## Metabolic reprogramming and plasticity

It has been shown that the epithelial-mesenchymal transition (EMT) can endow cancer cells with stem cell-like properties and can cause a switch from an epithelial program to a motile mesenchymal phenotype [48]. However, in solid tumors, CSCs can arise independently of EMT. A comparative analysis using metabolomic and fluxomic approaches identified metabolic profiles that differentiate metastatic prostate epithelial CSCs from non-CSCs expressing a stable EMT signature. The epithelial CSCs (ECSCs) are distinguished by an enhanced Warburg effect and a greater carbon and energy source flexibility resulting from amino acid and fatty acid metabolism. ECSCs are also characterized by a critical dependence on the proton buffering capacity bestowed by glutamine metabolism. A metabolic gene signature for ECSCs has been correlated with tumor progression and metastasis in several cancer types [45].

The induction of EMT is associated with enhanced glycolysis and reduced mitochondrial activity. Mechanistic analysis demonstrated that this process is the result of the activation of cytochrome c oxidase [49] or from the suppression of fructose-1,6-bisphosphatase [22]. Furthermore, bioenergetic disorders resulting from the inhibition of citrate synthase or succinate dehydrogenase subunit B can contribute to the acquisition of an EMT phenotype [50]. Luo et al. reported that EMT-driven CSCs can metabolize alternative high-energy metabolites, the phenomenon known as reverse Warburg effect (Table 1) [51].

The comparison between mesenchymal-like CSCs (MCSC) and ECSCs revealed distinct metabolic pathways. MCSCs display enhanced glycolysis as well as reduced O_2_ consumption, reduced ROS production, more antioxidant capacity, and reduced mitochondrial mass and membrane potential compared to ECSCs [30, 52]. Recent work has divided GSCs into two subtypes with a mesenchymal GSC population as the more malignant subtype. Glycolytic and Aldehyde dehydrogenase 1A3 (ALDH1A3) activities are remarkably elevated in mesenchymal GSCs but not in proneural GSCs. Moreover, irradiation of proneural GSCs results in an up-regulation of mesenchymal-associated markers and a down-regulation of proneural-associated markers, and this effect is attenuated by inhibition of ALDH1A3 activity. For the high-grade glioma patients with the mesenchymal signature, inhibition of ALDH1A3-mediated pathways is thus a promising therapeutic approach [53].

The article "Crosstalk between autophagy and metabolic regulation of cancer stem cells" was published in 2020. Journal: Mol Cancer.

Along the same line, Luo et al. also recently reported that proliferative ECSCs and quiescent MCSCs in breast cancer display different sensitivities to inhibitors of glycolysis and redox metabolism. Metabolic or oxidative stress promotes the transition of MCSCs with low levels of ROS to ECSCs with high levels of ROS. This transition depends on the AMPK-HIF1α pathway and is reversed by N-acetylcysteine. Moreover, silencing of expression of the gene encoding nuclear factor erythroid 2-like 2 (NRF2) or suppression of downstream thioredoxin and glutathione antioxidant pathways result in ECSCs sensitive to ROS-induced differentiation and cytotoxicity. However, both MCSCs and ECSCs are eliminated by co-inhibition of glycolysis and thioredoxin and glutathione pathways. This co-inhibition abolishes tumor-initiating potential, tumor growth, and metastasis [54]. The CSC phenotype is glycolytic in in vitro experiments, given the non-physiological concentrations of oxygen and glucose, whereas directly after cells are isolated from patients or after the first passage in culture CSCs depend on OXPHOS [52]. The upregulation of the glucose transporter Glut3 results in increased production of GSCs indicating how the high-grade glioblastomas, which are endowed with a high metabolic plasticity, survive in glucose-poor environments [55].

## Metabolism as a therapeutic target for CSC

Several pathways which regulate metabolism and autophagy of CSCs, are targeted for the treatment of cancer (Table 2 and Fig. 2). Anti-CSC therapies causing a deficiencies in energy and materials impairing CSC survival and propagation establish the basis of the future therapies. The following paragraphs provide a brief preview of these therapeutic target and the compounds that influence metabolism and autophagy of CSCs.

**Table 2:** Drugs targeting CSC metabolism

Metabolism-based strategies	Compound	Mechanism of action	CSC or tumor type	Reference
Glycolysis inhibition	2-Deoxy-D-glucose	Glycolysis inhibitor	Breast CSCs	[21]
	3-BP	Glycolysis inhibitor	Glioblastoma CSCs, PDACs	[56]
	DCA	Metabolic shift from glycolysis to OXPHOS	GBM cells	[57]
Inhibition of mitochondrial respiration	Metformin	Complex I inhibitor	Pancreatic CSCs, CSCs of HT29 cell line derived from colorectal cancer	[32, 58]
	Phenformin			
	Rotenone			
	Antimycin-A	Complex III inhibitor	Lung CSCs	[59–62]
	Bedaquiline	Complex V inhibitor	Breast CSCs	
	Oligomycin	Complex V inhibitor	Glioblastomas	
	Salinomycin analogs	Lysosomal iron sequestration	Breast CSCs	[63]
		Impairs autophagic flux	Breast CSCs	[64]
		Interference with ABC transporters	Breast, AML, lung, gastric, osteosarcoma, colorectal, pancreatic and prostate CSCs	[65]
		Activation of the Wnt/β-catenin signaling pathway		
	188Re-Liposome	Mitophagy inhibitor	Ovarian CSCs	[66]
	Doxycycline	Mitochondrial biogenesis inhibitor and inducer of apoptosis	Breast and cervical CSCs	[67, 68]
	XCT-790	ETC uncoupler, mitochondrial biogenesis inhibitor, inhibitor of ERRα-PGC-1 signaling pathway	Breast CSCs	[31]
	Mdivi-1	Fission inhibitor, inhibitor of assembly of Drp1 and its GTPase activity	Breast CSC, brain tumor initiating cells	[69, 70]
Redox homeostasis and antioxidant signaling	Zaprinast	Inhibition of glutathione biosynthesis, glutaminase inhibitor	Non-small lung and glutamine-addicted pancreatic cancer cell lines	[30, 59, 71]
	BPTES			
	968			
	BSO			
	Apigenin	Neutralizer of ROS-induced NRF2 activity, STAT3 signaling pathway inhibitor, inhibitor of the NRF2 and NF-ƙB pathways	Ovarian and prostate CSCs, triple-negative breast cancers, leukemia stem-like cells	[72–76]
	ATRA			
	Brusatol			
	Disulfiram			
	Trigonelline			
Lipid metabolism	2M14NQ	Blocks CD36 activity and fatty acid uptake	Glioblastoma CSCs	[77]
	Soraphen A	Inhibitor of ACC	Breast CSCs	[78–80]
	Chloroquine	Inhibition of autophagy	Breast CSCs	[15, 64]
	TVB-2640	FASN inhibitor	Breast CSCs	[78]
	MF-438	SCD-1 inhibitor, inhibitor of FAO	Lung CSCs, liver cancer, glioblastoma and AML cells	[81, 82]
	SSI-4			
	A939572			
	Etomoxir			
	ST1326	Inhibition of FAO	AML cells	[83, 84]
	Avocatin B			
	Emodin	ACLY inhibitor	Lung CSCs	[85]
	TVB-2640	Inhibitor of HMG-COAR, inhibitor of cholesterol synthesis through the mevalonate pathway	Breast and brain CSCs	[34, 86]

The article "Crosstalk between autophagy and metabolic regulation of cancer stem cells" was published in 2020. Journal: Mol Cancer.

**Fig. 2:** Metabolic modulators with anti-CSC effects. Metabolic pathways such those involving glutamine, glycolysis, redox balance, lipids, and autophagy are potentially targetable in CSCs. Some of the metabolic enzymes that are currently being considered as therapeutic targets for CSC are indicated by blue rectangles in the figure. Transcription factor NRF2 plays a pivotal role in both intrinsic resistance and cellular adaptation to ROS and is shown in a yellow rectangle. The carnitine-dependent transporter, which inhibits the mitochondrial import of fatty acids is shown in a yellow ball. Inhibitors are indicated by red rectangles. Abbreviations: ACC, acetyl-CoA carboxylase; Ac-CoA, acetyl-coenzyme A; ACLY, ATP citrate lyase; ACSL, long-chain acyl-CoA synthetases; ATRA, all-trans retinoic acid; 3-BP, 3- bromopyruvate; BSO, L-buthionine-S,R-sulfoximine; CPT1, carnitine palmitoyltransferase; I/Q/II/III/IV/V, complexes of the electron transport chain; DCA, dichloroacetate; 2-DG, 2-deoxy-D-glucose; Doc, doxycycline; FASN, fatty acid synthetase; FAT/CD36, Fatty acid translocase; GCS, gamma glutamyl cysteine synthetase; GLS, glutaminase; GLUT1/4, glucose transporter 1/4; GSH, glutathione; HK2, hexokinase 2; HMG-CoAR, 3-hydroxy-3-methyl-glutaryl-coenzyme A reductase; 2M14NQ, 2-methylthio-1,4-naphthoquinone; Mito, mitochondrial; NRF2, nuclear factor erythroid 2-related factor 2; OAA, oxaloacetate; PDH, pyruvate dehydrogenase; ROS, reactive oxygen species; TC, tetracyclines; TCA, tricarboxylic acid cycle; SCD1, stearoyl-CoA desaturase-1; SLC1A5, solute carrier family 1 member 5;

## Mitochondrial metabolism

As mentioned above, mitochondria play a key role in the responses to oxidative stress, energy status changes, and apoptotic stimuli and are also involved in the regulation of stemness and differentiation of CSCs [59]. Several pathways that promote anaerobic and aerobic energy metabolism of CSCs have been evaluated as targets for the treatment of cancer (Fig. 2).

### OXPHOS inhibitors

Various compounds that inhibit oxidative metabolism result in sensitization of CSCs to chemotherapies, leading to their eradication. This has been demonstrated in a model of PDAC. KRAS mutations are known to be a driver event of PDAC, but targeting mutant KRAS has proved challenging. Using a KRAS-inducible mouse model, Viale et al. demonstrated that a subpopulation of cells with CSC features survives KRAS-ablation therapy and induces tumor relapse [87]. Transcriptomic and metabolic analyses of surviving cells demonstrated a strong expression of genes driving mitochondrial function and lysosomal and autophagic activity as well as a robust dependence on mitochondrial respiration and a decreased dependence on glycolysis for cellular energetics. Importantly, these cells depend on OXPHOS for survival.

These CSC have high sensitivity to OXPHOS inhibitors and when OXPHOS inhibitors are combined with a targeted inhibitor of the KRAS pathway tumor recurrence is blocked [88]. However, metformin, which acts directly on the respiratory chain complex I in the mitochondria to inhibit OXPHOS and reduce mitochondrial ATP production (Fig. 2), was not enough to eliminate the CSC subpopulation [32]. This is possibly due to their intermediate glycolytic/respiratory phenotype and also to the heterogeneity and plasticity of PDAC cells. A previous study demonstrated that metformin increases ROS production in CSCs from PDAC cells and reduces their mitochondrial transmembrane potential. The AMPK/mTOR axis is not involved in the subsequent induction of lethal energy crisis in CSCs.

The article "Crosstalk between autophagy and metabolic regulation of cancer stem cells" was published in 2020. Journal: Mol Cancer.

Interestingly, Kim et al. recently demonstrated that glutamine metabolism also plays an important role in regulation of the sensitivity of colorectal CSCs to metformin through a mechanism that depends on the AMPK/mTOR pathway. In the absence of glutamine, but not in low-glucose medium, CSCs from SW620 cells were sensitive to the CSC-suppressing effect of metformin with activation of AMPK and suppression of mTOR. A combination of metformin and glutaminase C inhibitor compound 968, an inhibitor of glutamine metabolism, suppressed proliferation of CSCs in SW620 cells and enhanced the effect of metformin alone in HT29 cells (Fig. 2). Thus, the sensitivity to metformin in this cell line is possibly due to activation of AMPK pathway.

Depletion of alanine serine cysteine transporter 2 (ASCT2), glutaminase 1, and c-MYC induced significant CSC suppression. The compounds 968 and metformin also induced CSC elimination, and the activities were enhanced by silencing of *ASCT2* and *c-MYC*. Thus, the effect of metformin on CSCs varies depending on the extent of activation of the AMPK/mTOR pathway and glutamine metabolism [58]. Consistent with a metabolic profile dominated by OXPHOS, ovarian CSCs undergo apoptosis upon inhibition of the mitochondrial respiratory chain by oligomycin, antimycin, rotenone, and metformin (Fig. 2).

CSCs have higher mitochondrial ROS production and elevated membrane potential as well as enhanced pentose phosphate pathway activity compared to normal counterparts. This metabolic characteristic is not representative of cells that privilege OXPHOS over glycolysis and may instead reflect the role of the pentose phosphate pathway in reloading scavenging enzymes [29]. In agreement with this, combined treatment with 5-fluorouracil, an inhibitor of thymidine synthesis, and a pharmacological inhibitor of OXPHOS abolishes drug resistance of colon cancer cells in culture and diminishes the expression of stem-like markers [89].

The efficacy of metformin has prompted efforts to repurpose available drugs to target CSCs (for review see [59]). Various FDA-approved antibiotics known to target the mitochondrial respiratory chain have been shown to selectively decrease CSC survival or proliferation (Fig. 2 and Table 2). Examples are antimycin A, a powerful complex III inhibitor that decreases lung spheroids; the anti-tuberculosis agent bedaquiline (a complex V inhibitor) that inhibits mammosphere formation; oligomycin (another complex V inhibitor) that synergistically suppresses growth and motility of glioblastoma cell lines when combined with 2-deoxy-D-glucose (2-DG); and niclosamide, an anti-helminthic with OXPHOS uncoupling properties [90], that inhibits proliferation of CSCs from ovarian and breast cancers. Niclosamide also prevents the conversion of breast non-CSCs into CSCs induced by IL-6 [91]. Salinomycin also inhibits CSC formation in diverse cancer types [65]; OXPHOS is known to be inhibited by salinomycin [92]. Depletion of ATP levels and induction of mitophagy and mitoptosis are observed in cancer cells treated with salinomycin [93]. As a pleotropic compound that also interferes with Wnt signaling and ABC transporters, the antitumoral effect of salinomycin likely results from a combination of factors [65]. We recently demonstrated that salinomycin impairs autophagic flux [64] and kills CSCs by sequestering iron in lysosomes by ferroptosis [63] (Fig. 2).

The article "Crosstalk between autophagy and metabolic regulation of cancer stem cells" was published in 2020. Journal: Mol Cancer.

The compound known as XCT-790 also prevents breast CSC survival and propagation. The rescue of the effect of XCT-790 by acetyl-l-carnitine (a mitochondrial fuel) indicates that mitochondria are the target of XCT-790 in CSCs [31]. XCT-790 is a strong and selective inverse agonist ligand of the estrogen-related receptor alpha (ERRα), which is a cofactor of peroxisome proliferator-activated receptor gamma co-activator (PGC-1α). PGC-1α is the master regulator of mitochondrial biogenesis and is essential for the activation of numerous nuclear transcription factors that control the transcription of many mitochondrial genes [94]. Independent of its inhibition of ERRα and mitochondrial biogenesis, XCT-790 is a potent mitochondrial electron transport chain uncoupler [95] (Fig. 2).

Numerous classes of FDA-approved antibiotics also inhibit mitochondrial biogenesis to eliminate CSCs [96]. These include the erythromycins, the tetracyclines, the glycylcyclines, an anti-parasitic drug, and chloramphenicol. Efficacy was observed across eight different tumor types (breast, ductal carcinoma in situ, ovarian, prostate, lung, pancreatic, melanoma, and glioblastoma), suggesting that cancer can be treated as an infectious disease. Indeed, simultaneous inhibition of autophagy and treatment with antibiotics significantly reduces tumorigenic properties of cancer cells suggesting that this should be tested as a potential strategy for anticancer therapy [97]. However, continuous treatment with antibiotics for cancer therapy may not succeed due to induction of autophagy or a glycolytic shift.

The article "Crosstalk between autophagy and metabolic regulation of cancer stem cells" was published in 2020. Journal: Mol Cancer.

### Mitochondrial dynamics inhibitors

Mitochondria are dynamic organelles that often undergo fusion and fission events to sustain mitochondrial integrity and appropriate bioenergetics and spatial distribution. High levels of mitochondrial fission activity are associated with high proliferation and invasiveness in some cancer cells and with self-renewal and resistance to differentiation in some stem cells [98]. A specific inhibitor of the fission events, mDIVI1, induced apoptosis in brain tumor initiating cells and inhibited tumor growth. mDIVI1 is an inhibitor of dynamin-related protein 1 (DRP1), a mitochondrial fission protein, induces mitochondrial oxidative stress and reduces mitochondrial metabolism. CDK5-dependent DRP1 activation in brain tumor initiating cells stimulates mitochondrial fission preventing cell death and sustaining self-renewal and growth. DRP1 activation in brain tumor initiating cells correlates with poor glioblastoma patient survival [69]. Recently, Peiris-Pages et al. showed that mDIVI1 prevents breast CSC survival and propagation [70].

Mitochondrial fission can produce an impaired daughter unit that is targeted by the autophagic machinery. Mitochondrial fusion, on the other hand, may serve to dilute impaired respiratory components and thereby prevent their removal. The inverse dependency of fusion and mitophagy on membrane potential allows these two processes to act in a complementary rather than competitive fashion on the daughter mitochondrion after a fission event [99]. Intraperitoneal delivery of the nanomedicine 188Re-Liposome killed the CSCs-like cells in tumors with a degree of selectivity and switched metabolism from glycolysis to OXPHOS in an animal model of ovarian cancer [66] (Fig. 2). A study showed that dynamin 1-like -mediated mitochondrial fission induced by liensinine, a novel mitophagy inhibitor, sensitizes breast cancer cells to chemotherapy [100]. Recently, Chang et al. showed that mitophagy inhibitors such as liensinine and 188Re-Liposome abolish drug resistance in ovarian CSC-like cells [101].

### Glycolysis inhibitors

Previous findings suggest that CSCs may be specifically dependent on a high glucose turnover; therefore, targeting the glycolytic pathway is a promising therapeutic approach. Zhou et al. demonstrated that the combination of a glycolysis inhibitor such as 3-bromopyruvate (3-BP) with standard therapeutic agents such as doxorubicin killed glioblastoma CSCs and inhibited tumor formation. This study suggests that stem-like cancer cells prefer a low oxygen microenvironment and actively utilize the glycolytic pathway [18]. Recently, Isayev et al. showed that treatment with 3-bromopyruvate almost completely blocked cell viability, self-renewal potential, NF-κB binding activity, and stem cell-related signaling and reverted gemcitabine resistance of CSCs from PDAC [56].

The article "Crosstalk between autophagy and metabolic regulation of cancer stem cells" was published in 2020. Journal: Mol Cancer.

The switch from mitochondrial OXPHOS to cytoplasmic glycolysis is accompanied by development of the resistance to cell death in glioblastoma multiforme. This metabolic switch is accompanied by mitochondrial hyperpolarization. Michelakis et al. demonstrated that dichloroacetate (DCA), a small-molecule drug, induced a metabolic shift from glycolysis to OXPHOS, resulting in increased ROS, and induced apoptosis in CSC glioblastoma [57]. By inhibiting pyruvate dehydrogenase kinase (PDK), DCA activates PDH, increasing the ratio of glucose oxidation to glycolysis. On activation of PDH, however, pyruvate can be decarboxylated to acetyl-coenzyme A, enter the TCA cycle, and complete glucose oxidation in the mitochondrial matrix, generating up to 36 mol of ATP per glucose molecule in the presence of oxygen.

## Targeting redox homeostasis and antioxidant signaling

Growing evidence supports a model for redox homeostasis in which the ROS-antioxidant interaction acts as a metabolic interface for signals derived from metabolism and from the environment. This interface regulates processes that allow cells to acclimate or, alternatively, to die. The efficacy of clinically used classical chemo and radiotherapy is due to high levels of intracellular ROS-induced cancer cell death. However, Yuan et al. recently reported that ROS generated from OXPHOS is essential in CSC activation [102], which promotes tumor development. This suggests that high levels of ROS may not eradicate CSCs.

CSCs are characterized by a finely regulated redox metabolism [103]. Glutathione plays an essential role in maintenance of stemness characteristics [104]. Glutathione synthesis may be inhibited either directly or indirectly by blocking glutamine synthetase (GS) or glutaminase enzymes (GLS). Several glutaminase inhibitors have been evaluated preclinically [30], including buthionine sulfoximine (BSO), 968, and bis-2-(5-phenylacetamido-1,3,4-thiadiazol-2-yl) ethyl sulfide (BPTES) [59] (Fig. 2). Recently, zaprinast, an asthma medication was identified as a glutaminase inhibitor [71]. Depletion of glutathione and inhibition of thioredoxin reductase activity could also enhance radiation responses in human breast and pancreatic CSCs by a mechanism involving thiol-dependent oxidative stress. The following pharmacologically agents inhibit glutathione and thioredoxin metabolism: BSO; sulfasalazine (SSZ), an inhibitor of xc (−) cysteine/glutamate antiporter; auranofin, a thioredoxin reductase inhibitor; and 2-AAPA, a GSH-reductase inhibitor. Combined inhibition of glutathione- and thioredoxin-dependent thiol metabolism can enhance responses of CSC to conventional therapies [105].

The article "Crosstalk between autophagy and metabolic regulation of cancer stem cells" was published in 2020. Journal: Mol Cancer.

As mentioned above, NRF2 is a transcription factor that mediates the cytoprotective response to oxidative and electrophilic stress. Under the oxidative stress, NRF2 dissociates from its molecular inhibitor Kelch-like ECH-associating protein 1 (KEAP1) and translocates into the nucleus. There NRF2 binds to the antioxidant response element (ARE) of its target genes to induce their expression. NRF2 target genes include *NADPH quinone oxidoreductase-1* (*NQO-1*) and *aldo-keto reductase 1C1* and genes encoding glutathione generating enzymes and drug efflux transporters such as breast cancer resistance protein (BCRP). Recently, Kim et al. reported that all-trans retinoic acid (ATRA) inhibits NRF2 activation, suppresses ALDH1 expression, and leads to the attenuation of ovarian CSC-like properties [72] (Fig. 2).

In the presence of copper, administration of disulfiram, an approved anti-alcoholism drug, significantly downregulates ALDH1A1, CD44, and phospho-STAT3 levels. Disulfiram suppresses stem-like properties in triple-negative breast cancer by targeting the STAT3 signaling pathway [73]. Moreover, in leukemia stem-like cells, disulfiram and copper selectively activate the stress-related ROS-JNK pathway and simultaneously inactivate the NRF2 and NF-κB pathways [74]. Although disulfiram is now begin tested in phase III clinical trials, it is extremely unstable in blood. To increase disulfiram blood levels, a nanocarrier system of mPEG-PLGA/PCL has been used for the delivery [106].

Many other NRF2 inhibitors, including brusatol, apigenin, and trigonelline, have been identified (Fig. 2). Brusatol treatment suppresses NRF2 at the protein level, which results in enhanced intracellular ROS, sensitization of mammospheres to taxol, and reduced anchorage-independent growth. However, further studies are needed to establish its in vivo action. Apigenin [75] and trigonelline [76] are transcriptional and translational NRF2 inhibitors, respectively, that were developed as adjuvants to chemotherapeutic drugs. Mechanistic analyses demonstrated that *NRF2* silencing or treatment with trigonelline abolishes the ferroptosis resistance of KEAP1-deficient and cisplatin-resistant cancer cells to artesunate [76]. Paradoxically, some natural antioxidants, including sulforaphane, curcumin, resveratrol, oleanane triterpenoid, and carnosol, which all increase NRF2 expression levels, also have therapeutic potential. Readers interested in detailed discussion of this paradox should see recent reviews [59, 107].

The article "Crosstalk between autophagy and metabolic regulation of cancer stem cells" was published in 2020. Journal: Mol Cancer.

## Lipid metabolism

The role of lipid metabolism as a major source of energy and metabolic intermediates was recently demonstrated for processes implicated in transformation of normal cells into malignant cells and tumor progression [59]. Lipid metabolism is necessary for synthesis of membrane components. Fatty acids are broken down through mitochondria beta oxidation, which produces acetyl-coenzyme A (Ac-CoA) for anaplerosis. Citrate, a TCA cycle intermediate, can be used as a precursor for fatty acid synthesis and for NADPH production through the ATP citrate lyase (ACLY) (Fig. 2). Citrate is subsequently converted to acetyl-CoA and oxaloacetate in the cytoplasm. ACLY links glycolytic and lipidic metabolism. ACLY is overexpressed in cancer cells, and siRNA-mediated silencing of *ACLY* limits cancer cell proliferation and reduces the capacity of A549 lung cancer cells to form spheres [108]. ACLY inhibitors, previously developed for metabolic disorders, have recently attracted interest as promising anti-cancer agents [109]. Koerner et al. recently synthesized an emodin derivative and demonstrated that this novel ACLY inhibitor prevents proliferation of lung CSCs in vitro [85] (Fig. 2 and Table 2).

The committed step of fatty acid synthesis is the activation of acetyl-CoA to malonyl-CoA. This is an energy-consuming process catalyzed by acetyl-CoA carboxylase (ACC). The acetyl and malonyl groups are then coupled to the acyl-carrier protein domain of the multifunctional fatty acid synthase (FASN). Repeated condensations of acetyl groups generate the basic 16-carbon saturated palmitic acid. FASN activity is higher in adult murine neuronal stem and progenitor cells than in differentiated progeny [110]. Fatty acids are required for the production of phosphoglycerides, which, together with cholesterol, can be used for building cell membranes. Lipid droplets store triacyl glycerides and cholesteryl esters. Emerging data indicate that stored cholesteryl ester and accumulation of lipid droplets are correlated with tumorigenicity of CSCs derived from neurospheres and from ALDH^+^/CD133^+^ ovarian cancer cells [111] and colorectal cancer cells [112]. Thus, increased lipid storage in lipid droplets appears as a CSCs marker [112]. Lipids from extracellular sources can also be stored in lipid droplets. Thus, lipid metabolism is controlled by fatty acid synthesis and fatty acid oxidation (FAO) as well as by NADH, which is necessary for the production of ATP [113]. Lipolysis of lipids stored in lipid droplets was earlier considered to be solely carried out by cytosolic lipases. However, recent studies demonstrate that lipophagy (autophagic degradation of lipids by acidic lipases) serves as an alternate pathway for the degradation of lipid droplets [113]. Among target tested for CSC elimination, lipid metabolism is promising [59]. Several compounds that influence lipid metabolism have been tested preclinically (Fig. 2 and Table 2).

The article "Crosstalk between autophagy and metabolic regulation of cancer stem cells" was published in 2020. Journal: Mol Cancer.

### Lipid uptake inhibition

Lipid uptake can be inhibited by pharmacological inhibition or by antibody-mediated inhibition of the transporter fatty acid translocase CD36. Dietary lipid dependence of metastasis-initiating cells has recently been reported in melanoma and breast cancer. Inhibition of CD36, by specific antibodies, impairs metastasis [114]. Conversely, over-expression of CD36 significantly increases lymph node metastasis of oral squamous cell carcinoma cell lines with low metastatic potential [114]. Metastatic-initiating cells are also characterized by a distinct lipid metabolic signature related to fatty acid degradation, de novo lipogenesis, and lipid storage. CD36 is enriched in CSCs from glioblastoma and functionally distinguishes self-renewing cells. CD36 is co-expressed with integrin alpha 6 and CD133, previously described CSC markers, and CD36 reduction results in concomitant loss of integrin alpha 6 expression, self-renewal, and tumor initiation capacity. 2-Methylthio-1,4-naphtoquinone (2M14NQ), a unique sulfur-containing quinone, which inhibits CD36 activity, decreases self-renewal ability and induces apoptosis in glioblastoma CD133^+^ CSCs [77] (Fig. 2). CD36^+^ leukemia CSCs are enriched in gonadal adipose tissue and have elevated fatty acid uptake and beta oxidation [115]. Sulfosuccinimidyl oleate, another CD36 inhibitory compound, decreases proliferation of chemoresistant leukemic CD36^+^/CD34^+^ stem cells [115]. The conversion of long chain fatty acids to fatty acyl-CoAs is catalyzed by the long-chain acyl-CoA synthetases (ACSL), which have been linked to carcinogenesis [116]. The ACSL inhibitor triacsin C is under investigation for the treatment of acyl-CoA synthetase-dependent tumors. However, there is no data available on the ACSL as a therapeutic target for CSC.

### Inhibition of lipogenesis and acyl-CoA synthetase lipid desaturation: FASN and stearoyl-CoA desaturase-1

Results of a recent study support the theory of re-activation of de novo lipogenesis in solid tumors as part of cancer metabolic reprogramming [113]. In invasive ductal carcinoma, acetyl CoA synthetase 2 (ACSS2), an enzyme that catalyzes the conversion of acetate to acetyl CoA, is overexpressed under hypoxic and lipid-depleted conditions. ACSS2 increases acetate consumption and thereby fatty acid biosynthesis in the harsh tumor microenvironment where there is a scarcity of alternate carbon sources for lipogenesis. Thus, targeting de novo lipogenesis and lipid desaturation could provide a selective mechanism to interfere with tumor growth.

The article "Crosstalk between autophagy and metabolic regulation of cancer stem cells" was published in 2020. Journal: Mol Cancer.

A specific inhibitor of the first committed step of lipid biosynthesis catalyzed by ACC, the antifungal polyketide soraphen A, suppresses growth of breast CSCs [78] (Fig. 2 and Table 2). Numerous classes of ACC inhibitors have been evaluated in clinical trials for metabolic diseases (i.e., obesity and metabolic syndrome). Mechanistic analysis suggests that the biotin carboxylase domain of the ACC, which is the soraphen A binding subunit dimerization site, may be an ideal target for ACC inhibitors with potential for use in cancer therapy.

#### FASN inhibitors

Given the involvement of the enzyme FASN in numerous tumor types, FASN inhibitors including C75, C93, epigallocatechin gallate, G28UCM, orlistat, Fasnall, GSK2194069, and GSK837149A have been evaluated in a mouse model of breast cancer [79]. Inhibition of FASN by cerulenin and of mevalonate pathways by atorvastatin prevents proliferation of CSCs in vitro [80] (Fig. 2 and Table 2). C75 at non-cytotoxic concentrations significantly reduces the capacity of MCF-7/HER2 cells to form mammospheres, an in vitro indicator of cancer stem-like cells [117]. Despite these efforts, however, the majority of FASN inhibitors have failed to advance into clinical trials due to unexpected toxicities. Currently, TVB-2640 is the only selective FASN inhibitor in clinical trials for the treatment of advanced solid tumors, including HER2^+^ advanced breast cancer, high-grade astrocytoma, colon cancer, and non-small cell lung carcinoma with mutations in KRAS.

#### SCD1 inhibitors

A recent report using hyperspectral-stimulated Raman spectroscopic imaging and mass spectrometry analysis of extracted lipids showed that ovarian CSCs contain unusually high levels of unsaturated fatty acids (UFAs) and that UFAs are essential for the cells to retain stemness. These data suggest that increases in lipid unsaturation might be a general marker for CSCs in ovarian cancer and a new target for CSC-specific therapy [118]. Stearoyl-CoA desaturase-1 (SCD1), the most abundant desaturase, is expressed in lipogenic tissues and catalyzes the formation of double bonds at the ninth carbon atom of saturated fatty acids, leading to mono-unsaturated fatty acids. Using molecular approaches and chemical inhibitors such as CAY 10566 and SC26196, SCD1 was identified as the enzyme responsible for the increased desaturation in stem cells. Mechanistically, UFAs increase NF-κB activity, which upregulates expression of *ALDHA1* and *SCD-1* mRNAs. Increased SCD1 in turn promotes UFA synthesis from saturated fatty acids, forming a positive feedback loop [118].

The article "Crosstalk between autophagy and metabolic regulation of cancer stem cells" was published in 2020. Journal: Mol Cancer.

Two studies support the use of combination therapy with SCD1 inhibitors to achieve better control of cancer [81]. The first study reported that SCD1-mediated endoplasmic reticulum stress regulates liver tumor-initiating cells and sorafenib sensitivity. SCD1 inhibitors A939572 or SSI-4 alone or in combination with sorafenib thus have potential for treatment liver cancer [81]. In parallel, Pisnau et al. reported that co-treatment with cisplatin and the SCD1 inhibitor MF-438 decreases expression of lung CSCs markers, strongly synergizes in the inhibition of sphere formation, and induces apoptosis of lung CSCs [82] (Fig. 2 and Table 2). However, clinical utilization of SCD1 inhibitors for anti-cancer therapy should proceed with extreme caution. SCD1 is also involved in the regulation of inflammation and stress in various cell types, including β-cells, adipocytes, macrophages, endothelial cells, and myocytes.

Considering the established link between obesity and risk for many types of cancer, the observation that SCD1 deficiency protects mice against high-fat diet-induced obesity and hepatic steatosis [119] suggests that SCD1 inhibitors could serve the dual purpose of blunting tumor growth and preventing obesity and associated metabolic conditions. On the other hand, loss of SCD1 function is associated with the development of inflammatory diseases such as dermatitis, atherosclerosis, intestinal colitis, pancreatic β-cell dysfunction, and liver dysfunction [119]. Furthermore, SCD1 is highly expressed in the brain. Small-molecule inhibitors of SCD1 could cross the blood-brain barrier and interfere with the axon myelination process. Therefore, therapeutic strategies that target the re-activation of de novo lipogenesis of tumor tissues should take into consideration the risks of interference with active de novo lipogenesis in normal tissues.

### Inhibition of fatty acid oxidation

FAO is a promising target for elimination of CSCs. Etomoxir, an inhibitor of the carnitine-dependent transporter CPT1 (also known as CPT1A), which inhibits the mitochondrial import of fatty acids mediated by the carnitine shuttle, decreases intracellular ATP levels as well as the viability and resistance to chemotherapy of glioblastoma and acute myeloid leukemia cells [120]. Silencing of *Nanog* or overexpression of cytochrome c oxidase subunit 6A and/or inhibition of FAO by etomoxir, sensitizes CSCs to sorafenib treatment. These data suggest that FAO inhibition or OXPHOS reestablishment to induce metabolic reprogramming of CSCs should be a powerful therapy in hepatocellular carcinoma [121]. Unfortunately, the clinical development of etomoxir was terminated because of severe hepatotoxicity and hematopoietic stem cell exhaustion associated with treatment [120]. However, alternative FAO inhibitors are under investigation. For instance, the compound ST1326 strongly inhibits chemoresistance of leukemia cells with no effect on normal stem cells [83]. Additionally, another FAO inhibitor, avocatin B, which acts as a lipid that accumulates in mitochondria, eliminates CSCs from acute myeloid leukemia with no effect on normal blood stem cells [84] (Fig. 2 and Table 2).

The article "Crosstalk between autophagy and metabolic regulation of cancer stem cells" was published in 2020. Journal: Mol Cancer.

### Cholesterol synthesis through the mevalonate pathway

Cholesterol synthesis from acetyl-CoA proceeds through the mevalonate pathway. Analysis of a large cohort of breast cancer patients provided evidence of reduced mortality in statin users. Statins are inhibitors of 3-hydroxy-3 methylglutaryl-CoA reductase (HMG-COAR), the limiting step of the mevalonate pathway. However, these associations are weak in magnitude and attenuated in some sensitivity analyses [122]. As mentioned above, treatment with various statins targeting CSC self-renewal resulted in elimination of CSCs in breast [34] and brain [86] cancers. Moreover, a mixture of brutieridin and melitidin, which has statin-like properties, eradicates CSCs by targeting mevalonate, Rho-GDI-signaling, and mitochondrial metabolism [123]. In addition, bergamot metabolically inhibits OXPHOS and FAO [123].

## Concluding remarks

It is now clear that the cancer is a heterogeneous disease and that metabolic heterogeneity and flexibility of tumor cells contributes to this heterogeneity. Location influences CSC metabolic status. In actively growing regions of the tumor and in the presence of adequate levels of oxygen, CSCs rely on glycolytic and/or oxidative metabolism. In nutrient-poor states, autophagy is activated as an alternative energy source. The catabolic glycolysis/oxidative phosphorylation and the anabolic gluconeogenesis pathway control glucose homeostasis. The metabolic adaptation of CSCs to the tumor microenvironment may provide an explanation for the metabolic differences observed in CSCs. However, further investigation are necessary to demonstrate the role of autophagy in plasticity and metabolic reprogramming. Current studies have revealed details of CSC metabolism in terms of redox state, lipid metabolism, and use of alternative fuels, such as amino acids or ketone bodies, identifying important vulnerabilities that could provide new therapeutic opportunities. However, to interrogate the metabolic traits of CSCs, metabolism must be analyzed directly after isolation from patients or after very few passages in culture to avoid artifactual switches in metabolic characteristics.

The article "Crosstalk between autophagy and metabolic regulation of cancer stem cells" was published in 2020. Journal: Mol Cancer.

## Data Availability

Not applicable.

## Abbreviations

2-DG: 2-deoxy-D-glucose
2M14NQ: 2-methylthio-1,4-naphtoquinone
3-BP: 3- bromopyruvate
ACC: Acetyl-CoA carboxylase
Ac-CoA: Acetyl-coenzyme A
ACLY: ATP citrate lyase
ACSL: Long-chain acyl-CoA synthetases
ACSS2: Acetyl CoA synthetase 2
ALDH1A3: Aldehyde dehydrogenase 1A3
AMPK: AMP-activated protein kinase
ARE: Antioxidant response element
ASCT2: Alanine serine cysteine transporter 2
ATP: Adenosine triphosphate
ATRA: All-trans retinoic acid
BCRP: Breast cancer resistance protein
BCSCs: Breast cancer stem cells
Bnip3: Bcl-2/adenovirus E1B interacting protein 3
BPTES: Bis-2-(5-phenylacetamido-1,3,4-thiadiazol-2-yl) ethyl sulfide
BSO: L-buthionine-S,R-sulfoximine
CAFs: Cancer-associated fibroblasts
CPT1: Carnitine palmitoyltransferase
CS: Citrate synthase
CSC: Cancer stem cell
DCA: Dichloroacetate
DNMT: DNA methyltransferases
Doc: Doxycycline
DRP1: Dynamin-related protein 1
ECSCs: Epithelial CSCs
EMT: Epithelial-mesenchymal transition
ERRα: Estrogen-related receptor alpha
F6P: Fructose-6-phosphate
FAO: Fatty acid oxidation
FASN: Fatty acid synthetase
FAT/CD36: Fatty acid translocase
FBP1: Fructose-1,6-biphosphatase
FOXO3A: Forkhead box 3A
G6PDH: Glucose-6-phosphate dehydrogenase
GBM: Glioblastoma
GCS: Gamma-glutamylcysteine synthetase
GDH: Glutamate dehydrogenase
GFAT: Glutamine-fructose-6-phosphate transaminase 1
GLS: Glutaminase
GLS1: Mitochondrial glutaminase
GLS2: Cytosolic isoform glutaminase
GLUT1, 2, 3, 4: Glucose transporter 1,2, 3,4
GS: Glutamine synthetase
GSC: Glioblastoma stem cells
GSH: Glutathione
HIF-1α: Hypoxia-inducible factor 1α
HK2: Hexokinase 2
HMG-CoAR: 3-hydroxy-3-methyl-glutaryl-coenzyme A reductase
I/Q/II/III/IV/V: Complexes of the electron transport chain
JNK/AP1: c-Jun N-terminal kinases/activator protein 1
KEAP1: Kelch-like ECH-associating protein 1
KLF4: Kruppel-like Factor 4
LC3: Microtubule-associated Protein 1 Light Chain 3
LDH: Lactate dehydrogenase
MCSC: Mesenchymal-like CSCs
MCT2/4: Monocarboxylate transporter 2/4
Mito: Mitochontrial
NADH: Nicotinamide adenine dinucleotide (reduced)
NADPH: Nicotinamide adenine dinucleotide phosphate (reduced)
NAMPT: Nicotinamide phosphoribosyl transferase
NANOG: Nanog Homeobox
NF-κB: Nuclear factor-κB
NMN: Nicotinamide mononucleotide
NNMT: Nicotinamide N-methyltransferase
NQO-1: NADPH quinone oxidoreductase-1
NRF2: Nuclear factor erythroid 2–related factor 2
OAA: Oxaloacetate
OCT4: Octamer-binding transcription factor 4
OXPHOS: Oxidative phosphorylation
P: Phosphate (or phospho)
PARPs: Poly (ADP-ribose) polymerases
PDAC: Pancreatic ductal adenocarcinoma
PDH: Pyruvate dehydrogenase
PDK1: Pyruvate dehydrogenase kinase 1
PFKFB: Phosphofructokinase/fructose bisphosphate
PGC-1α: Peroxisome proliferator-activated receptor gamma co-activator
PHGDH: Phosphoglycerate dehydrogenase
PKM2: Pyruvate kinase isozyme M2
RHOA: Homolog family member
ROS: Reactive oxygen species
SAM: S-adenosyl methionine
SCD1: Stearoyl-CoA desaturase-1
SFA: Saturated fatty acids
SIRTs: Sirtuins
SLC1A5: Solute carrier family 1 member 5
SOX2: Sex determining region Y-box 2 S
SZ: Sulfasalazine
TC: Tetracyclines
TCA: Tricarboxylic acid cycle
TGF-β: Transforming growth factor β
UFA: Unsaturated fatty acids.

The article "Crosstalk between autophagy and metabolic regulation of cancer stem cells" was published in 2020. Journal: Mol Cancer.

## Glossary

Electron transport chain: A series of transmembrane protein complexes, present on the inner membrane of mitochondria, that transfer electrons via redox reactions to the terminal electron acceptor oxygen, which is reduced by binding of protons to a water molecule. This generates a proton gradient that powers ATP synthase to produce ATP. Premature leakage of electrons to oxygen can lead to production of reactive oxygen species.
Anaplerosis: The act of replenishing TCA cycle intermediates used for macromolecule biosynthesis.
Cataplerosis: The removal of intermediate metabolites, especially those resulting from the TCA cycle, to prevent their accumulation in the mitochondrial matrix.
Glutathione: A tripeptide (glutamate-cysteine-glycine) that acts as an important antioxidant. The reduced form of glutathione can react with H_2_O_2_ to form the oxidized form (GSSG).
Glutaminolysis: A series of biochemical reactions by which the glutamine is lysed to generate molecules such as CO_2_, alanine, aspartate, citrate, glutamate, lactate, and pyruvate. When glycolytic energy production is low, glutamine, the most common amino acid in the plasma, serves as an additional energy source for tumor cells. Glutamine is also a nitrogen source for amino acids, hexosamines (amino sugars involved in the synthesis of glycosylated molecules), and nucleotides. In cancer cells, glutamine metabolism fuels the TCA cycle, fatty acid and nucleotide biosynthesis, and redox balance. Most cancer cells consume glutamine, and many tumors are thought to be addicted to glutamine [124]. This addiction results largely from the contribution of glutamine to anaplerosis [125].
Macroautophagy: Referred to here as autophagy, allows the orderly degradation of cellular components and recycling of amino acids, lipids, nucleic acids, and saccharides from intracellular nutrient stores. In this catabolic process, double-membraned vesicles called autophagosomes form around cellular cargo, including organelles, protein aggregates, and intracellular pathogens. After fusion of autophagosome with a lysosome, the cargo is degraded.
Nicotinamide adenine dinucleotide (NAD) metabolism: NAD acts as an electron and hydrogen acceptor during glycolysis, fatty acid oxidation, and the TCA cycle. NAD also serves as a coenzyme for oxidoreductases and dehydrogenases that generate ATP during nutrient degradation, playing a key role in cellular respiration. NAD and its phosphorylated and reduced forms, including NADP, NADH, and NADPH, are essential for cell metabolism activities. NAD most often functions in catabolic energy-generating reactions where it is reduced to NADH. The phosphorylated form, NADPH, participates in anabolic reactions, such as the synthesis of fatty acids and cholesterol. In addition to its function in oxidative phosphorylation and redox reactions, NAD is a substrate for evolutionarily conserved NAD cleavage enzymes such as poly (ADP-ribose) polymerases (PARPs), sirtuins (SIRTs), and cADP-ribose synthases such as CD38 and CD157.
